RETRACTED

# Construction of a Health Management Model for Early Identification of Ischaemic Stroke in Cloud Computing

**DOI:** 10.1155/2022/1018056

**Published:** 2022-03-22

**Authors:** Yuying Yang, Qing Chang, Jing Chen, Xiangkun Zhou, Qian Xue, Aixia Song

**Affiliations:** ^1^Stroke Center Office, The First Affiliated Hospital of Hebei North University, Zhangjiakou, Hebei 075000, China; ^2^Department of Neurology, The First Affiliated Hospital of Hebei North University, Zhangjiakou, Hebei 075000, China; ^3^Imaging Department, The First Affiliated Hospital of Hebei North University, Zhangjiakou, Hebei 075000, China; ^4^Information Section, The First Affiliated Hospital of Hebei North University, Zhangjiakou, Hebei 075000, China

## Abstract

Knowledge discovery and cloud computing can help early identification of ischaemic stroke and provide intelligent, humane, and preventive healthcare services for patients at high risk of stroke. This study proposes constructing a health management model for early identification and warning of ischaemic stroke based on IoT and cloud computing, and discusses its connotation, constructive ideas, and research content so as to provide reference for its health management in order to develop and implement countermeasures and to compare the awareness of early stroke symptoms and first aid knowledge among stroke patients and their families before and after the activity. The rate of awareness of early symptoms and first aid among stroke patients and their families increased from 36% to 78%, and the difference was statistically significant (*P* < 0.05) before and after the activity.

## 1. Introduction

A health education team was formed in the Department of Emergency Medicine and the Department of Neurology to promote early symptom recognition and first aid knowledge, and a clear division of labour and standardised teaching materials created a good space and atmosphere for teaching [1–3]. In addition, the “Green Health” WeChat public number was set up to promote stroke and first aid knowledge through the Internet in the form of graphics and videos, which not only enriched the form of education on stroke disease and first aid knowledge but also broadened the publicity channels and helped to promote the education of stroke patients and their families on stroke disease and first aid knowledge. This is conducive to the homogenisation of stroke patients' and families' knowledge of stroke disease and first aid, and can improve the effectiveness of education [4–6].

Using WeChat as a new communication medium not only breaks the limits of time and space but also allows for the instant dissemination of new knowledge and information, enabling interactive communication between healthcare professionals and patients and their families [3] so that stroke patients and their families can learn about stroke disease knowledge and first aid anytime and anywhere, thus increasing the level of knowledge of stroke disease and first aid among patients and their families [7].

RETRACTED

Quality management is an automatic and spontaneous activity carried out by people at the work site or in interrelated areas [8], characterised by a combination of leaders, technicians, and employees, with individuals gaining a sense of involvement and achievement in their work [9]. At the same time, circle activities improve the motivation of the circle members, enhance team cohesion, and contribute to the progress and development of the stroke patient team. Therefore, quality management circle activities can improve the work ability of individual members and promote the development of stroke patient teams [10].

In summary, the use of quality management circles not only improves the ability of stroke patients and their families to identify early symptoms but also gives full play to the individual potential of the circle members, improves their individual work ability, and promotes the development of the stroke patient workforce.

## 2. Stroke Management Model

### 2.1. Internet of Things

The IoT management model is based on Internet of Things (IoT) technology and with its superior bionic characteristics. It is a powerful tool in expanding human thinking, liberating human labour, and promoting social progress. In summary, the IoT management model is a four-sided linkage of the sensing side (radio frequency identification, sensors, etc.) [11], the transmission side (Internet, mobile Internet and 5G technology, etc.) [1], the cloud side (cloud computing, big data technology, artificial intelligence, etc.), [12] and the application side (various network platforms), with each side integrating technological innovation, management innovation, and institutional innovation, forming a modern intelligent management model of “four linked ends and three in one” [13].

The sending end is the base layer of the IoT management model and is the necessary gateway for the exchange of information in the virtual and real space of the IoT management model [14]. In other words, the sensing side is the input side of the IoT management model system, which acts directly on the environment, and the information technology mainly relies on its various sensing devices that identify and capture information, such as radio frequency identification (RFID) technology and wearable devices.

The cloud is the “brain” of the IoT management model, relying on powerful comprehensive analysis functions to continuously output power for the survival of the IoT management model [15]. After receiving the information captured by the sensing end, the cloud uses modern information technology, such as big data technology and management cloud computing, to conduct a comprehensive analysis. This process takes decision makers out of the tedious process of information analysis and allows them to focus on making good decisions [16].

RETRACTED

The “trinity” innovation system of the IoT management model, with its “four-end linkage” organisational structure, only provides a realistic framework for the IoT management model, but to make it work in practice, it is necessary to rely on the “trinity” system. “Trinity” system guarantees to clear the realistic obstacles for the IoT management model [17–19].

### 2.2. Health Management

Health management is a process of comprehensive management of health risk factors for an individual or a population [20]. This process is carried out by professionals who provide advisory guidance and follow-up counselling services to enable individuals to receive comprehensive health maintenance and protection services in multiple dimensions, including social, psychological, environmental, nutritional, and exercise, through health information collection, health testing, health assessment, personalised health management programmes, and health interventions [21].

## 3. Building Ideas

Data collection: patients at a risk of stroke have their signs collected by lower limb muscle monitors, voice recognition devices, and other sign monitoring devices [22]. Operation and monitoring: the data are transmitted wirelessly to the user's terminal access device and application software, and the stroke cloud platform organises it into a database for monitoring, calculation, and analysis. Once the monitored indicators reach the threshold, an alarm signal will be sent out via GPS and healthcare professionals will take immediate action to ensure that the stroke patient is treated within a short and valuable window of time (see Figure 1).

To achieve partial encryption of medical stroke patient privacy information based on cloud computing, a data transfer model for encrypting medical stroke patient privacy information is constructed in a finite domain [23]. The ciphertext transfer protocol is Decrypt (sk, *c*^*∗*^)*A*^−1^=*T*=(*t*_*i*,*j*_)_*i*,*j*=1_^*m*^, the encrypted transfer control of the medical stroke patient privacy information system is performed using public key cryptography, the system master key is constructed, and the dynamic key for encrypting medical stroke patient privacy information safely is as follows:

(1) $$\begin{array}{c} TA=\left(t_{1,1},\ldots ,t_{m,m}\right)\left(a_{1,1},\ldots ,a_{m,m}\right). \end{array}$$

Using the security parameter *ν* as input, the unscripted data in the medical stroke patient privacy information are authorized to be encrypted using a random variable signed encryption algorithm, a user authentication protocol for encrypting medical stroke patient privacy information is established, and an encapsulation protocol for partially encrypting medical stroke patient privacy information is constructed [24], and the entropy and minimum entropy for encrypting medical stroke patient privacy information are obtained as shown in equation (2), respectively.

(2) $$\begin{array}{c} \text{Decrypt }\left(\text{sk},c^{*}\right)A\left(\alpha_{1},\ldots ,\alpha_{m}\right){\left(A^{-1}\right)}^{{\left(\alpha_{1}^{-1},\ldots ,\alpha_{m}^{-1}\right)}^{\text{T}}}\\ =\left(\alpha_{1}^{-1}t_{1,1},\ldots ,\alpha_{m}^{-1}t_{m,m}\right)\left(\alpha_{1}a_{1,1},\ldots \alpha_{m}a_{m,m}\right)\\ =E. \end{array}$$

For the identity user, considering the randomness of the output certificate, the security parameter K and symmetric key K of medical stroke patient privacy information encryption are input, and the key of medical stroke patient privacy information system encryption is reset. Through the key expansion method, the key expansion sequence *X*=*x*_1_, *x*_2_,…, *x*_*n*_ of medical stroke patient privacy information is obtained. The method of p-order cyclic group mapping is adopted. The weighted vectors ${\overset{⟶}{s}}_{i,j}^{\left(0\right)}$ and ${\overset{⟶}{s}}_{i,j}^{\left(1\right)}$ of medical stroke patients' privacy information with a length of $\sqrt{\Theta }$ bits are generated, and the encrypted ciphertext sequence of medical stroke patients' privacy information is *S*_*n*_=*x*_1_+, *x*_2_+⋯+*x*_*n*_. The user *ID*_*i*_ and message *M* are entered, and the ciphertext of layer *L*+1 of medical stroke patients' privacy information transmission data is shown in the following equation:

(3) $$\begin{array}{c} \mathrm{Decrypt}\;\left(\text{sk},c^{*}\right)AA^{-1}=\left(t_{1,1},\ldots ,t_{m,m}\right)=E. \end{array}$$

Using the keyword encryption algorithm, the user *ID*_*i*_ private key *sk*_*ID*_*i*__ and two identities *ID*_*i*_, *ID*_*j*_ are entered and the output sequence of plaintext medical stroke patient privacy information is as follows:

(4) $$\begin{array}{c} \text{Decrypt }\left(\text{sk, }c^{*}\right){\left[A\left(\alpha_{1},\cdots ,\alpha_{m}\right)\right]}^{-1}=\left(\;\right.\begin{array}{ccc} \alpha_{1}^{-1} & t_{1,1}, & \cdots ,\\ \alpha_{m}^{-1}t_{m,m} & =\left(A^{-1}\right){\left(\alpha_{1}^{-1},\ldots ,\alpha_{m}^{-1}\right)}^{\text{T}}. & \; \end{array} \end{array}$$

The resulting arithmetic coding model for encrypting private information of medical stroke patients is shown in Figure 2.

RETRACTED

This paper proposes a cloud-based data encryption algorithm for establishing an arithmetic coding model for stroke patient privacy information and designing a key for stroke patient privacy information [25].

(5) $$\begin{array}{c} P-\text{value }=2+\frac{1}{\varphi \left(S_{\text{obs}}\right)}\\ =2+\left(1-2\pi \sum_{-\infty }^{\text{Sobs}}{\text{e}}^{-2u^{2}}\right)=3-2\pi \sum_{-\infty }^{\text{Sobs}}{\text{e}}^{-2u^{2}}. \end{array}$$

The decrypted private key of *ID*_*i*_ is used for key resigning to obtain a statistic *P* value ≥ 0.01 for the decrypted key, and the transformed ciphertext is processed for cloud information fusion when it satisfies *KS* ∈ {0,1}, by generating four empty lists *H*_1_ − list, *H*_2_ − list, *ds*  *k* − list, and *rsk* − list to obtain a linear encoding distribution function for the privacy information of medical stroke patients, as shown in the following equation:

(6) $$\begin{array}{c} f^{-1}\left(I\right)=\left\{\begin{array}{cc} p+I, & s=0,\\ \frac{1}{\left(1+p\right)*I}, & s=1, \end{array}\right. \end{array}$$

where Ι denotes the private key of the medical care private message sender; the initial value I = [0, 1] is set, *f* is rewritten as *f*(*y*)=∑_*i*=0_^*q*_*H*_^*c*_*i*_*y*^*i*^ to obtain the feature vector *v* ∈ *Z*^*μ*×*μ*^, the public key of the medical care private message transmission *pk*=*se*_2_, (*u*_*i*,*j*_)_1≤*i*,*j*≤*μ*_,  *se*_3_,  (*δ*_*i*_^(0)^)_0≤*i*_,  (*δ*_*i*_^(1)^)_0≤*i*_ private key *sk*=(*s*_*i*_, *s*_*i*,*j*_)1 ≤ *i*, *j* ≤ *μ* is calculated to obtain the medical stroke patient privacy information encryption and decryption protocol [24, 26].

*h*_1_′,…, *h*_*q*_′ ∈ *Z*_*p*_1__^*∗*^ is randomly selected to achieve key construction of private information for medical stroke patients, as shown in Figure 3.

## 4. Case Studies

### 4.1. Object

110 stroke patients and their families in the Emergency Medicine and Neurology Departments from 18 March 2020 to 18 April 2020 were selected for the preprotocol circle activity, and 110 stroke patients and their families hospitalized from 25 April 2020 to 25 June 2020 were selected for the postprotocol circle activity.

Stroke patients and their families have little knowledge of stroke risk factors and early warning signs, with a 23.7% awareness rate of stroke warning signs [27]. The majority of stroke patients in China do not recognise stroke symptoms at an early stage thus delaying the best time for treatment, which seriously affects the outcome and prognosis of stroke patients. Therefore, the theme of this campaign is to raise awareness of early warning for stroke patients and their families so as to improve their ability to recognise stroke symptoms and knowledge of first aid and to enable them to seek timely medical attention and receive effective treatment [28].

RETRACTED

### 4.2. Results

After the implementation of the campaign, the awareness rate of patients and family members about early stroke symptoms and first aid was 78%, based on the formula: target achievement rate = (postimprovement data - preimprovement data)/(target value - preimprovement data) × 100%, resulting in a target achievement rate of 116.7%. Knowledge of early stroke symptoms and first aid among stroke patients and their families before and after the event is shown in Table 1.

The circle members have grown in the use of QC techniques, team spirit, responsibility and honour, communication and coordination, motivation, logical thinking, professional knowledge, and personal potential, especially in the area of QC techniques and personal potential (see Figure 4).

## 5. Simulation Test Analysis

MATLAB was used to design the experiments. The key extraction homomorphic vector was $\left.O\left(\gamma +\left(\beta +\sqrt{\Theta }\right)\left(\mu^{2}.\eta +\lambda \right)\right)=O\left(\lambda^{5.5}\right)\right)=25$, and the sampling frequency of the private information of stroke patients was 15 MHz Table 2.

Based on the above parameter settings, the partial encryption of private information of medical stroke patients was obtained, and the time-domain distribution of the original encrypted data was obtained [29, 30], as shown in Figure 5.

Using the data in Figure 5 as the study object, the partial encryption of stroke patients' private information was performed and the encryption results were obtained, as shown in Figure 6.

Analysis of Figure 6 shows that the method in this paper can effectively achieve the partial encryption of private information of medical stroke patients, with good encryption resistance to attacks. The encryption depth was tested, and the comparison results were obtained, as shown in Table 3.

As can be seen from Table 3, when the number of iterations is 100, 200, 300, 400, etc., the test results obtained by using this paper for the encryption depth of medical stroke patients' privacy information are higher than those obtained by traditional methods, and when the number of iterations is 400, the encryption depth of medical stroke patients' privacy information by using this paper is as high as 400 dB. The encryption is more resistant to attacks, and the encryption depth is deeper.

## 6. Conclusions

The incidence of stroke is currently high, but the state of implementation of early stroke recognition is worrying. The delay in admission of stroke patients is serious, with a delay in the attendance rate of approximately 60%. The early identification of ischaemic stroke patients needs urgent improvement. The application of this model, consisting of muscle force acquisition sensors, voice acquisition sensors, network data storage, cloud data processing, mobile cloud clients, and network transmission, can achieve accurate and timely identification of ischaemic stroke patients who have just developed a stroke at any time and any place, and provide timely alerts through Internet of Things and cloud platform [29, 30].

RETRACTED

## Figures and Tables

**Figure 1:** IoT and cloud-based health management model for early identification and warning of ischaemic stroke.

**Figure 2:** Arithmetic coding model for encryption of private information of medical stroke patients.

**Figure 3:** Key design for private information of medical stroke patients.

**Figure 4:** Five star result radar map.

**Figure 5:** Time-domain distribution of data encryption.

**Figure 6:** Encrypted data output.

**Table 1:** Comparison of stroke patients' and families' knowledge of early stroke symptom recognition and first aid.

Time	Number of people	Know (person)	Awareness rate (%)
Before development	110	40	36
After development	110	86	78

**Table 2:** Experimental parameter settings.

Parameter setting	*t*_max_	M	L	*P*_*m*_	*P*_*c*_
Parameter value	12	26	13	0.45	0.79

**Table 3:** Medical stroke patient privacy information encryption depth test.

Iterations (time)	This method/dB	Reference [4] (dB)	Reference [5] (dB)
100	13.57	8.21	11.76
200	24.75	11.46	13.54
300	32.44	15.53	22.53
400	42.65	20.46	25.57

## Data Availability

The authors did not obtain analytical permission from the data provider because of trade confidentiality.
